# Effect of chemical disinfection on the dimensional stability of polyvinyl ether siloxane impression material: a systemic review and meta-analysis

**DOI:** 10.1186/s12903-023-03168-8

**Published:** 2023-07-10

**Authors:** Saeed Awod Bin Hassan, Abdulkhaliq Ali F Alshadidi, Lujain Ibrahim N Aldosari, Artak Heboyan, Ravinder S Saini

**Affiliations:** 1 Department of Restorative Dental Sciences “RDS” College of Dentistry, King Khalid University, Abha, Kingdom of Saudi Arabia; 2 Deptt. Dental Technology, College of Medical Applied Sciences, King Khalid University, Abha, Saudi Arabia; 3 Prosthodontics Department, College of Dentistry, King Khalid University, Abha, Saudi Arabia; 4 Department of Prosthodontics, Faculty of Stomatology, Yerevan State Medical University after Mkhitar Heratsi, Str. Koryun 2, Yerevan, 0025 Armenia; 5 Deptt. Dental Technology COAMS, King Khalid University, Abha, 62529 Kingdom of Saudi Arabia

**Keywords:** Vinyl polyether siloxane, PVES, Hybrid elastomeric impression material, Chemical disinfection, Sodium hypochlorite, Glutaraldehyde

## Abstract

**Background and objectives:**

Polyvinyl ether siloxane (PVES) possesses ideal characteristics for making precise and accurate dental impressions. PVES dimensional stability owes to its better polymeric properties derived from its parent materials poly ethers and polyvinyl siloxanes. As recommended use of chemical disinfecting agents is getting more popular, there is a growing concern associated with the effect of disinfectants on PVES dimensional stability. This study was aimed to understand the PVES behavior when subjected to chemical disinfectants.

**Materials and methodology:**

The data was collected from research studies retrieved from Google Scholar, Scopus, and PubMed using MeSH terms of keywords “vinyl polyether siloxane AND Disinfection” or (Vinyl polyether siloxane OR polyvinyl siloxane ether OR PVES) AND (disinfectant OR disinfection)” without any restriction to publication date. The PRISMA (Preferred Reporting Items for Systemic Review and Meta-Analysis) directions were observed during the data collection, screening of studies, and meta-analysis. The primary data were retrieved, and batch exported from databases using Harzing’s Publish or Perish software; primary analysis was performed in Microsoft Excel, while statistical analysis for effect size, two-tailed p-values, and heterogeneity among studies was performed using Meta Essentials. The effect size was calculated using Hedge’s g values at the 95% confidence level using the random-effects model. Heterogeneity among studies was measured using the Cochrane Q and I^2^.

**Results and conclusion:**

Dental impressions made from the PVES elastomeric impression materials showed no significant changes in dimensional stability. Immersion in the chemical disinfectant for 10 min was associated with clinically irrelevant changes in the dimensions of the PVES impressions. Disinfection with sodium hypochlorite was associated with clinically significant changes in dimensions, with a two-tailed p-value of 0.049. Disinfection with 2–2.5% glutaraldehyde solution was not associated with any significant dimensional variability.

**Supplementary Information:**

The online version contains supplementary material available at 10.1186/s12903-023-03168-8.

## Introduction

Perfect restoration in dentistry often corresponds to a meticulous and precise impression. However, it is challenging for many clinicians and technicians to obtain an impression of fixed prostheses. Clinicians strive to maintain the accuracy and reproduction of dental impressions by selecting reliable impression materials from a plethora of materials. Elastomeric materials provide a combination of physical and chemical properties that are often enjoyed by clinicians and technicians. One emerging elastomeric material is vinyl polyether siloxane (PVES), a hybrid of polyether (PE) and polyvinyl siloxane (PVS) [1, 2]. This reinvigorated elastomeric polymer combines the dimensional accuracy of polyvinyl silanes with the hydrophilic properties of polyether [3]. PVES is claiming a fair share in restorative dentistry owing to its desirable features that are well-suited for making impressions in dental prostheses.

A PVES hybrid is an elastomeric impression material that possesses good physicochemical properties and surface characteristics inherited from those of PE and PVS. It has better wettability and better mechanical and flow characteristics and is available in low-, medium-, and high-body viscosities. It is well established that impressions made from PVES are accurate for finer details on wet dental surfaces or in the gingival sulcus [4, 5]. Although the accuracy of impressions is often implied by the polymeric characteristics of the elastomers, other factors that can impact the impressions are clinical and technical factors. Technical factors include impression trays and techniques, whereas clinical factors include mandibular deformation, disinfection methods, and the chemical nature of disinfectants.

### Impact of disinfectants on dental impressions

Dental impressions, including those of PVES, come into contact with body fluids such as saliva and blood during the procedure. This poses the risk of contamination of master stone casts with infectious diseases, especially AIDS, hepatitis B, tuberculosis, and herpes simplex, as well as other opportunistic pathogens that can be fatal in immunocompromised patients [6–8]. Disinfection is recommended to avoid cross-contamination and remove bacteria, viruses, and other microorganisms. Commonly employed disinfecting agents include perchlorates and hypochlorites, iodophors, phenol, ethanol, isopropanol, and glutaraldehyde, which can disinfect microbes and spores using the spray method or immersion method [9].

Disinfectants are sprayed on the stone casts and impressions during spray disinfection. It is a rapid process, economical, and uses less disinfectant, which is significantly important when disinfecting colloids and polyether. However, this method does not provide satisfactory access to hard-to-reach areas of impression, such as undercuts. Aerosols produced during the process pose health risks to practitioners. However, the immersion method requires submerging the impressions into disinfectant solutions for a certain period of time to completely remove microorganisms [10]. It is time-consuming and requires the preparation of a fresh disinfectant for each use, which is discarded after a single use (excluding glutaraldehyde). Autoclaving, microwaving, irradiation with UV or gamma rays, and pasteurization are some of the less frequently practiced disinfection procedures [11].

Ideally, disinfectants should not interfere with the physical or chemical properties of the impression material, retaining the impression accuracy during the process [12]. The impression accuracy is attributed to the surface properties of the impression materials, such as dimensional stability, surface roughness, hydrophilicity, and detailed reproduction. Minute changes in these surface properties may lead to discrepancies in impressions, resulting in poor implants that slowly break down under chewing pressure. Clinicians prefer marginal gaps < 150 μm [13]. As the accuracy of impression and disinfection procedures goes hand in hand in dentistry, it is imperative to establish a standard disinfection procedure for specific impression materials. The accuracy of the impression can also be influenced by time, water content, temperature, and disinfection method (immersion or spray). Thus, procedures followed for the disinfection of impression materials as well as the chemical nature of disinfectants are significant contributing factors for making accurate dental impressions, and they need to be optimized for individual disinfectant–impression pairs.

Elastomeric impression materials, including PVES, are prone to shrinkage after removal, which becomes more pronounced with time, as the water content evaporates [14]. In contrast, disinfectant type and chemical nature may result in water imbibition, resulting in compromised accuracy. In the immersion method, impressions are submerged in a disinfectant for up to 30 min, providing sufficient time for hydrophilic elastomeric impression materials to absorb significant amounts of water [15, 16]. Several studies have reported that water content from disinfectants does not change the dimensional stability and accuracy of impressions, while others claim significant changes in dimensional stability with results that may or may not contribute to clinically significant dimensional changes.

This study is aimed to better understand the effect of disinfectants on the physical properties of vinyl polyether siloxane elastomers, including dimensional stability and surface quality. The research was designed on the hypothesis that the disinfectants which do not chemically react with the VPES material should not induce any changes in polymerized impressions during the disinfection process.

## Materials and methods

### Permission and registration

The framework of this systematic review was constructed based on the guidelines set out in the Preferred Reporting Items for Systematic Reviews and Meta-Analyses (PRISMA) [16]. The protocol used for this systematic review was the registered International Platform of Registered Systematic Review and Meta-analysis Protocols (INPLASY) (202,350,042).

The Preferred Reporting Items for Systemic Review and Meta-analysis (PRISMA) guidelines were kept in mind while searching and selecting research studies [17]. Databases such as Google Scholar, PubMed, and Scopus were systematically researched for relevant studies describing the effect of disinfection on the vinyl polyether siloxane using Boolean “AND” and “OR” terms along with medical search heading (MeSH) terms. The PICOS strategy consisted of the population – vinyl polyether siloxane, intervention – disinfection, control – native vinyl polyether siloxane, outcome – effect on accuracy of the dental impression, and source of study – in vitro studies. Research studies conducted until June 6th 2023, were included.

### Search strategy

Keywords for search terms were (vinyl polyether siloxane OR polyvinyl siloxane ether OR PVES) AND (disinfectant OR disinfection). Chemical disinfection was the procedure of interest, and a research query for systemic review and meta-analysis was designed accordingly. The main query was “Does chemical disinfection effects the accuracy and dimensional stability of the dental impressions made from PVES elastomers?” with the sub query “Are disinfectant induced changes in accuracy and dimensional stability of the PVES are clinically significant?”. The keywords and search terms used are listed in Table 1.

**Table 1:** Search terms used for extraction of research studies from databases

Boolean Search Strategies	
1.	Vinyl polyether siloxane AND Disinfection
2.	(Vinyl polyether siloxane OR poly vinyl siloxane ether OR PVES) AND (disinfectant OR disinfection)
3.	1 & 2

Studies were screened for inclusion and exclusion criteria by two independent researchers SH and LD. A third researcher, RS, was consulted to resolve any disputes regarding the inclusion or exclusion of studies. The included studies were included without any restrictions on the publication year. All in vitro studies with data on the effects of disinfection on PVES were included. Studies were selected based on the following criteria: [1] studies should have comparison data between native and disinfected PVES impressions, [2] methods of disinfection should be chemical disinfectants, and [3] studies published in English.

Initial screening for the eligibility of studies was performed using the title and abstract. Any ambiguity in the abstract or title was resolved by turning to a full-text article. Studies were then scrutinized through secondary screening by taking up the full text for disinfection procedures, data availability, PVES impression material, and sample sizes. Finally, the selected studies were used for a systemic review and statistical analysis.

### Exclusion criteria

Studies that did not provide any statistical data were excluded. Conference abstracts with comparison data between the native and disinfected dimensional accuracy of PVES were excluded. Clinical trials, these documents, survey reports, systematic reviews, and research studies published in languages other than English were also excluded. Studies were rejected if the comparison data were available without standard deviation, standard error, or mean standard error. Studies were also excluded if data were provided as percentages and non-standard forms, or data without sample size. Studies that used autoclaving, sterilization, irradiation, or any other non-chemical disinfection procedure were not considered due to lack of sufficient statistical data for meta-analysis.

### Data extraction

Studies were batch exported to MS Excel 2021 edition (Microsoft Corporation, Washington, USA) from corresponding research databases using Harzing’s Publish or Perish software (Tamra Software Research Limited) and GUI v8.8 Windows edition using Boolean terms and Mesh keywords. Extracted data contained information such as the title of research studies, year of publication, abstract, author names, no. of citations, type of publication, publication source and link to the original article, citations per year, and GS Rank. The final catalog of systemized studies included author names, title, and abstracts, publication year, disinfection procedure, accuracy of PVES impression in native form and with disinfection, dimensional accuracy of impression after exposure to chemical disinfectants, sample size, and statistical data. Data on dimensional discrepancies in PVES impressions along with immersion or spray disinfection methods were collected. Time-dependent changes in the accuracy of PVES impressions were also considered.

### Data analysis

Descriptive statistical analysis of the research data was carried out using MS Excel 2021 (Microsoft Corporation, Redmond, Washington, USA), and meta-analysis was performed using Meta-Essentials 2017 [17]. Impression accuracy and dimensional stability were compared for statistical analysis. The standard deviation (SD), standard mean differences, and pooled standard errors of the studies were calculated for meta–analysis, and effect size calculations. A two-tailed p-test was used to determine any significant correlation between the use of disinfectants and the resultant discrepancies in impression dimensional stability and accuracy. A p-value < 0.05 was deemed statistically significant for the p-test. Considering the differences in making impressions using various casting techniques, the standard error was calculated and used for further statistical analysis.

Effect size and meta-analysis were performed with 95% confidence intervals. The effect size was measured using a random-effects model and presented in ascending order. Heterogeneity was measured using the Cochrane Q and I^2^ to determine the extent of variance among the selected studies.

### Risk of bias analysis

Risk of bias analysis was done using Robvis Cochrane Risk of Bias analysis tool [18] due to invitro nature of studies. The studies were assessed on the basis of factors that can potentially affect the outcome of the study. The factors included were the control group, multiple measurements, bias in the outcome, bias in reporting results, and bias due to disinfection procedures. Each study was then assigned an overall score for risk of bias on these criteria. Each study was independently assessed by individual research for risk of bias.

## Results

### Studies included in systemic review

Studies included in this systematic review were searched in electronic databases as latest as 6th June 2023, which reported the effect of chemical disinfection on the dimensional accuracy of PVES elastomeric impression materials. The general depiction of the selection procedure is shown in the PRISMA flowchart in Fig. 1. A total of 362 studies were identified through automated database search, of which 305 were retrieved from Google Scholar, 12 from Scopus, and 45 from PubMed. After removing 33 duplicates, 329 studies underwent initial scrutiny for eligibility based on title and a short abstract. A total of 120 studies mentioned the keyword disinfection’ along with the terms’ polyvinyl siloxane ether’ or ‘vinyl siloxane poly ether’ or ‘vinyl siloxane ether’ in dental impression synthesis. After careful inspection during the secondary screening process, 20 studies were selected for the full-text analysis. The final screening of full-text articles put together 5 eligible articles, 13 studies did not meet the selection criteria or had inconclusive data to be included in the meta-analysis. One study reported the effect of disinfection on surface roughness only and was removed, and one reported on tear strength. One study was found through a manual search of citations. Finally, 6 studies were selected for the meta-analysis and systematic reviews. The detailed characteristics of the studies is shown in Table 2.

**Fig. 1:** PRISMA flow diagram for research studies included in this meta-analysis and systemic review

### Data extracted from the studies

The data extracted from the reported studies were the type of disinfection as spray or immersion method, while the chemical disinfectants employed for the process were recorded as glutaraldehyde, sodium hypochlorite (NaOCl), Dettol, Silosept, and Cavex. The data for dimensional stability measurement were either provided as the mean of dimensional changes before and after measurement or recorded from the values of the F-test and t-test on the experimental samples. Data regarding the time for disinfection, the amount of disinfectant used, and the number of samples used for the control and experimental groups were also collected to calculate the effect size. Data regarding comparative disinfection procedures using physical methods such as microwave or UV radiations were also collected but not used in this study.

### Effect of disinfection on dimensional stability

Data analysis revealed that the immersion method was the most commonly used disinfection procedure for PVES, with only one study reporting spray disinfection along with this immersion method. Almost all studies used a disinfection time of 10 min for the immersion method, only one study reported 30 min for glutaraldehyde disinfectant, and one study reported 3 min of disinfection for Cavex disinfectant. The results of the meta-analysis showed that the effect of chemical disinfection on the dimensional stability of PVES was insignificant. The immersion method used for disinfection of PVES may induce clinically acceptable minuscule changes. The results were supported by a two-tailed test with a p value above the significance threshold (p = 0.185). The data were considerably heterogeneous, with a Cochrane Q value of 37.75 and I2 value of 78.8%. Each study contributed almost equally to the cumulative effect size by weight (%). The meta-analysis was performed using a random effects model with values from Hedge’s g values at 95% confidence intervals of the upper and lower limits. The results of meta-analysis are depicted in Fig. 2.

**Fig. 2:** Meta-analysis results for the effect of immersion disinfection procedure on dimensional stability of PVES impressions

### Effect of glutaraldehyde and sodium hypochlorite on dimensional stability

Among disinfectants, glutaraldehyde and sodium hypochlorite (NaOCl) are the most commonly used disinfectants for immersion. The glutaraldehyde concentrations used ranged from 2 to 2.45%, whereas NaOCl concentrations ranged from 3 to 5.25%. It is worth noting that the overall effect of disinfection may be negligible, but the NaOCl disinfection method was associated with slightly higher alterations in VPES materials as compared to PE and VPS controls with a two-tailed test p-value of 0.049, though overall dimensional changes in VPES were not clinically significant.

**Table 2:** List of publication selected for this meta-analysis and systemic review along with respectively reported results for effect of disinfection on the dimensional accuracy of PVES impression material

Study	Material		Disinfectant composition		Disinfection method		Properties studied		Measurement specifications		Outcome		Limitations	
Khatri et al. 2020 (19)	PVES EXA’lence (GC Dental Products Corp, Japan) light and heavy medium		Glutaraldehyde 2.45% (Johnson and Johnson, India)		Immersed for 15 min		Linear dimensional stability		Dimensional changes recorded with Digital Vernier calliper under a stereomicroscope, measured at 0 h		Dimensional changes were within clinically acceptable range		The impressions were made from standard dies which do not resemble oral conditions	
			NaOCl 3.0% (Vishal, India)		Immersed for 15 min									
Mikaeel and Mustafa 2019 (20)	VPES (material brand and viscosity information not provided)		NaOCl 5.25%		Sprayed for 15 s and then left for 10 min, Immersed for 10 min		Linear dimensional stability, surface details		USB digital microscope, changes recorded after 7 and 48 h of disinfection		No significant dimensional difference in PVES after 7 h but clinically significant changes after 48 h		In vitro conditions, different time for disinfection for NaOCl and Dettol as compared to Cavex Impersafe	
			Dettol		Sprayed for 15 s and then left for 10 min, Immersed for 10 min									
			Cavex Impersafe		Sprayed for 15 s and then left for 3 min, Immersed for 3 min									
Mohd et al. 2021 (21)		VPES (Identium® (Kettenbach GmbH & Co. KG, Eschenburg, Germany), Medium body		Silosept® (Kettenbach GmbH & Co. KG, Eschenburg, Germany)		Immersed in disinfectant for 10 min, Rinse with water for 15 s		Linear dimensional stability		Dimensional changes recorded with Image Analyzer (Infinite Focus Real 3D Alicona), measured at 0 h		No significant Dimensional accuracy alterations for PVES		The dimensional accuracy of PVES was compared with PVS but not PE
Nassar et al. 2017 (22)	VPES EXA’lence (GC America Alsip, IL, USA). Heavy, light, and extra light consistencies with regular or fast set		Buffered Glutaraldehyde 2.5% (Metricide 28; Metricide Research, Orange, CA, USA)		Disinfected by immersion for 30 min under room temperature, rinsed for 15 s with water.		Linear dimensional stability		A milling machine. with an X and Y table and digital encoder with a resolution of 5 µ, aligned with a toolmaker microscope with 30X magnification. Measurements were taken at 0, 7 & 14 days.		No significant changes after 0 and 7 days while changes after 14 days were statistically significant.		Single disinfectant, disinfection duration of only one duration. Only VPES materials of different consistencies were compared, a better comparison would be with other impression materials like PE and PVS.	
Nassar and Chow 2015(23)	VPES EXA’lence (lot number 1,103,211; GC America, Alsip, IL). Heavy body, fast set.		Buffered Glutaraldehyde 2.5% (Metricide 28; Metricide Research, Orange, CA, USA)		Immersed for 30 min at room temperature, rinsed with water for 15 s.		Linear dimensional stability, surface details		A milling machine. with an X and Y table and digital encoder with a resolution of 5 µ, aligned with a toolmaker microscope with 30X magnification. Measurements were taken at 0, 7 & 14 days.		The material remained stable over the period of 14 days. VPES showed more stability as compared to VPS.		In vitro conditions	
Soganci et al. 2018 (24)	VPES EXA’lence (370 monophase, GC America, Alsip, IL, USA)		Glutaraldehyde 2.0% (Steranios, Anios Laboratoires, Hellemmes, France)		Immersed in disinfected for 10 min		3D dimensional stability		Dimensional changes recorded with 3D scanner (SmartOptics Activity 880, smart optics Sensortechnik, Bochum, Germany) at room temperature at 0 and 24 h after disinfection.		No significant effect on the dimensional accuracy of PVES		In vitro settings, the master model and conditions did not resemble the resiliency of oral tissues and saliva.	
			NaOCl 5.25% (Aklar Kimya, Ankara, Turkey)		Immersed in disinfected for 10 min									

The data heterogeneity for the glutaraldehyde-based disinfection process was very high, with an I2 value of up to 93% and a Cochrane Q value of 32.59. In the case of NaOCl based disinfection process, the data did not show heterogeneity at all with I2 values of 0.00 and Cochrane Q test value of 0.59, indicating consistency among research studies on NaOCl disinfection procedure. The effect size was calculated from Hedge’s g values using the random-effects model. The results are shown in Fig. 3.

**Fig. 3:** Meta-analysis results for the effect of glutaraldehyde and NaOCl on the dimensional stability of PVES impressions

### Quality and risk of bias

Robvis Cochrane Risk of Bias analysis (Fig. 4) showed one study [19] with high risk bias due to missing data on control groups and bias arising from longer than usual immersio method for disinfection. Two studies showed some conerns in risk of bias due to measurement of outcome [20] missing details on material properties [21]. Three studies showe lower risk of bias and were compliant with most of the factors used to measure the risk of bias. Hence, overall quality of studies showed low risk of bias in measurements and quality was deemed good for meta-analysis.

**Fig. 4:** Risk of bias analysis of studies included in this meta-analysis and systemic review

## Discussion

This study aimed to address the issue of using chemical disinfectants on PVES elastomeric impression materials and the resulting changes in dimensional accuracy during the preparation of dental impressions. This study is the first comprehensive report detailing effects of disinfection on the vinyl polyether siloxane. There was no systematic reviews and meta-analysis published on this topic till 6th June 9, 2023, to the best of our knowledge.

This meta-analysis and systemic review focused on the immersion method of disinfection using glutaraldehyde and NaOCl at different concentrations. Being hydrophilic, it is generally normal for elastomeric impression materials to absorb saliva and oral pathogens when preparing dental impressions in clinical practice. Gums are also prone to bleeding during the dental examination as well as impression making, and hydrophilic elastomers like PVES can absorb both saliva and blood during the process [9, 12, 22]. This makes the use of disinfectants mandatory to avoid any potential transmission of infectious agents among patients and clinicians alike. However, it is also necessary to resolve any speculations associated with the use of chemical disinfectants that affect the accuracy and stability of dental impressions.

According to the American Dental Association (ADA), dimensional changes below 0.5% (or below 20 μm) are considered within an acceptable range [23]. The PVES dimensions remained within a given range after disinfection. PVES is a hybrid material of polyether and polyvinyl siloxanes, which also demonstrates a great deal of dimensional stability when exposed to chemical disinfectants [24]. However, it is worth mentioning that in vitro research studies do not completely replicate the clinical conditions in which dentists use different types of adhesives, tray materials, and dental dies for dental impressions. Most studies also measured linear dimensional changes instead of more accurate three-dimensional measurements for dimensional accuracy.

The choice of disinfection method among dental practitioners may also vary depending on the choice of disinfectant and the clinical setup. Spray disinfection is generally considered to be a less effective control of pathogen count on dental impressions, whereas the immersion method is speculated to induce more dimensional changes. However, the results showed no significant difference in the dimensions of elastomeric impression materials when spray or immersion methods of disinfection were compared [25]. This study included data on both spray and immersion disinfection methods, which are commonly used by researchers. Only one study has compared the effect of spray disinfection in parallel with the immersion method using glutaraldehyde, Cavex Impersafe, and Dettol as disinfectants [20]. The use of 10 min of disinfection by submerging the PVES impressions or spraying with glutaraldehyde and Dettol did not result in significant dimensional alterations. The time used for Cavex was 3 min for both spray and immersion disinfection without any difference in the results.

Sodium hypochlorite and glutaraldehyde are commonly used for disinfection by immersion. NaOCl induced more dimensional changes in PVES than glutaraldehyde. Although the overall results for immersion disinfection showed no significant effect on dimensional variations, NaOCl-mediated disinfection was associated with significant dimensional variability in PVES impressions, as shown in Fig. 3. Although it is important to consider immersion time when calculating disinfectant-induced dimensional redoing, it is also important to consider how long after the measurements were taken. If measurements were taken long after the disinfection procedure, then alterations could occur due to the longer storage period, which is also known to be associated with dimensional changes irrespective of dimensional changes [26–28]. Storage time affects the water content of elastomeric polymers, and a significant amount of water is lost during long-term storage, resulting in shrinkage and dimensional changes in the dental impressions. For an accurate outcome, the significant impact of the storage period should not overlap with that of the disinfection period. This meta-analysis was based on data collected for the immersion period but did not have enough data available to carry out further analysis on dimensional transfiguration on storage and disinfection combined. Further analysis of the data on this subject is recommended for a clear understanding of the impact of disinfection on elastomeric impression materials.

The appropriate concentration for sodium hypochlorite to carry out impactful disinfection and negotiate with dimensional variabilities was 5.25% [20, 29]. However, Khatri M et al. [30] reported significant dimensional changes at 3% NaOCl concentration using the same duration for immersion disinfection. The resultant dimensional changes may have contributed to the waiting period after disinfection when measuring the dimensions of the immersion or post-disinfection treatment. For glutaraldehyde, 2–2.5% disinfectant concentration was safe enough to accomplish disinfection without significant consequences on the dimensional stability of the PVES impressions [29–31]. The meta-analysis results showed that this concentration of glutaraldehyde was not linked to the dimensional instability of the PVES material after immersion for 10 min. Although the results are not large enough to draw general conclusions, it shows that glutaraldehyde could be a cheaper and more effective disinfectant under dental clinical conditions to carry out disinfection on elastomeric impression materials in general, especially for PVES. Further research on this topic will provide a clearer understanding.

Almost all studies used 10 min of disinfection using glutaraldehyde and NaOCl as disinfectants, except one, which used 30 min of immersion time for glutaraldehyde immersion for PVES impressions. For commercial disinfectants, an immersion time of 10 min was used for Silosept and 3 min for Cavex disinfectants. There were not enough data to compare the significant impact of time duration on the dimensional stability of PVES impressions. From the available data, 30 min of immersion time for glutaraldehyde may have been a contributing factor to the dimensional changes in PVES [31]. However, data from published studies regarding other elastomeric impression materials indicate that immersion time has no clinically significant impact on the dimensional changes of dental impressions; rather, it is the type of solution used for immersion of dental prosthetic material [16]. Generally, silicon-based impression materials are more resistant to immersion disinfection than polyethers. Because PVES is a hybrid of silicones and polyethers, it is possible that different types of immersion solutions, rather than disinfectants, can harm the dimensional integrity of PVES dental impressions. There was not enough evidence to account for the composition of the disinfecting solution in the meta-analysis.

PVES disinfection is an important step in dental prostheses and prosthodontics to eliminate the potential threat of indirect transmission of infectious diseases. This meta-analysis and systematic review provide an overview of the current research on new hybrid PVES materials. The limitation of this study is the lack of data from the control group measurements; rather, it is derived from the dimensions of either die stones or master mold. Data are also limited in terms of the type of disinfectant and disinfection time for the PVES material. More research will provide a thorough understanding of PVES behavior under disinfectant chemical insults. In a broader context, other disinfecting procedures, including physical means such as UV and microwave radiation, autoclaving, or washing with ozonated water, should also be explored for PVES disinfection while preparing dental impressions.

Limitations of this study are those of type of disinfectants as data was only available for glutaraldehyde and sodium hypochlorite for VPES material and the effect of other disinfectants such as hydrogen peroxide, ozone, phenols, chlorhexidine, and other commercially available disinfectants could not be evaluated in context of dimensional reliability of VPES. Similarly, effect of spray disinfectants was only available for one study [20] and further research data in this regard will provide valuable information. This study was limited in discussing only dimension stability of the VPES and post-disinfection data for other physical properties such as surface details, elasticity, and tensile strength was not available. Some articles would have missed due to language limitations as well.

## Conclusion

This systematic review and meta-analysis is a headway to understanding PVES dimensional stability in the ever-evolving field of dental impressions and prosthodontics. It is fair to conclude from the published data that the currently employed disinfection procedures do not affect the dimensional stability of PVES impressions. Slight changes below 0.5% in dimensions during immersion disinfection were clinically insignificant. Considering the type of disinfectant, glutaraldehyde was least disruptive to dimensional stability with no significant effect on changes as compared sodium hypochlorite, albeit over dimensional discrepancies in either case were not clinically significant.

Disinfection of dental impressions is included in the Centers for Disease Control (CDC) recommendations as well as in clinical best practices to prevent any cross-contamination of dental impressions with potential infectious pathogens. This study provides a more detailed overview of the research conducted to date in this regard. The results showed that glutaraldehyde and sodium hypochlorite are the best choice as a disinfectant that effectively removes pathogens without any significant dimensional instabilities in PVES impressions.

## Electronic supplementary material

Below is the link to the electronic supplementary material.

Supplementary Material 1

Supplementary Material 2

Supplementary Material 3

Supplementary Material 4

## Data Availability

The datasets used and/or analyzed during the current study available from the corresponding author on reasonable request.
